# Knowledge about Hepatitis B Virus and Relevant Safety Precautions among Dental Students in Kurdistan Region, Iraq

**DOI:** 10.1155/2022/8516944

**Published:** 2022-09-18

**Authors:** Fadil Abdullah Kareem, Rahel Farhad Mohammad, Faraedon Mostafa Zardawi, Sarhang Sarwat Gul

**Affiliations:** ^1^Department of Pedodontics, Orthodontics and Preventive Dentistry, College of Dentistry, University of Sulaimani, Sulaymaniyah, Iraq; ^2^Periodontics Department, College of Dentistry, University of Sulaimani, Sulaymaniyah, Iraq

## Abstract

**Background:**

Hepatitis B virus (HBV) is still a major health problem worldwide, placing healthcare workers, medical and dental students, and professionals at higher occupational risk. The present study aimed to evaluate the level of knowledge about this virus and relevant safety precautions among dental students in the Kurdistan region of Iraq. *Materials and methods*. This cross-sectional study was conducted among the third, fourth, and fifth stage dental students of Hawler Medical, Sulaimani, and Duhok universities. Data on the students' demographic characteristics and their knowledge about HBV (16 close-ended questions) and safety precaution measures (10 close-ended questions) were collected by means of a questionnaire. Analysis of variance was used to compare the mean of knowledge and safety precaution scores.

**Results:**

In total, 372 students (mean age 21.77 ± 1.31 years) completed the questionnaires. The mean scores for knowledge and safety precautions were 13.17 ± 2.09 and 8.05 ± 1.61, respectively. Respondents from Hawler Medical University showed statistically significantly higher knowledge levels than their counterparts in Sulaimani and Duhok universities (*p* = 0.012).

**Conclusions:**

The majority of surveyed dental students are aware of HBV, its mode of transmission, infection, complications, vaccination, and safety precautions required to prevent the spreading of the virus. While the levels of knowledge about HBV and safety precautions among the dental students in the Kurdistan region of Iraq were generally acceptable, differences in knowledge level were identified between the universities, and these may be related to their educational and training programs.

## 1. Introduction

Hepatitis B virus (HBV) is classified as a DNA virus within the virus family Hepadnaviridae. Humans are regarded as the only known natural host. It circulates in the blood in concentrations as high as 108 virions per mm [1]. The virus has partially double-stranded DNA and a core antigen surrounded by a shell containing hepatitis B surface antigen which is considered the main diagnostic antigen for infection [2].

Replication of HBV happens only in the hepatic tissue. During high viral replication activity, the blood of an infected person may contain 106-1010 international units per mm, and, consequently, mucosal or parenteral contact with even a small amount of blood or body fluid may cause infection in susceptible people [3]. Annually, there are more than 50 million cases of acute HBV infections [4], with 5-10% of adults and up to 90% of infants suffering chronic infection [5]. Hepatitis B virus is considered to be the tenth leading cause of death throughout the world, and 500,000 to 1.2 million deaths per year are due to chronic hepatitis, cirrhosis, or hepatocellular carcinoma [4]. Iraq, meanwhile, is regarded to be of moderate endemicity for HBV infection, with a rate of 3% [6].

Transmission of infection in the dental practice might happen via infected needle prick, direct blood contact, saliva, and indirect contact with contaminated operative instruments or environmental surfaces [7], which can be prevented through the standard precautions adopted by the United States Centers for Disease Control and Prevention in 1996 [8]. These preventive measures must be followed by the dentist and dental team to overcome the risk of cross-infection. Moreover, the wearing of gloves by dentists and dental assistants has been recommended as a paramount component of cross-infection control [9].

Today, with the emergence and spread of the COVID-19, 6,454,184 of the world population were killed by the disease [10]. A dentist can play a crucial part in the prevention of hepatitis as well as COVID-19 infections by taking into account that each and every patient may be a potential carrier of hepatitis and COVID-19. Proper infection control measures, sterilization, and prophylactic vaccination protocols must be followed in order to minimize the risk of HBV infection, on the one hand [11], while ensuring dental care providers having a high level of knowledge is very important for their adoption of appropriate attitudes and practices regarding patients with HBV, on the other hand [12].

Accordingly, the dental staff's and dental students' knowledge and attitude are the cornerstones in the prevention of HBV infection. They are involved at the first stage of the dental health delivery system, and their coming into contact with infected patients and contaminated instruments might increase the risk of HBV and COVID-19 transmission, particularly if safety precautions are not followed correctly. As there is a lack of data on the awareness and practice among dental students in the Kurdistan region of Iraq, the purpose of the current study was to evaluate the knowledge and practice behavior of dental students, with a special focus on infection control and safety precautions that ultimately minimize transmission of this communicable disease, as well as to compare the knowledge and safety precautions regarding HBV infection among different dental colleges in the Kurdistan region of Iraq.

## 2. Materials and Methods

This cross-sectional study was conducted among the third, fourth, and fifth stage dental students of Hawler Medical, Sulaimani, and Duhok universities in the Iraqi Kurdistan region. The total numbers of dental students at these three universities were as follows: Hawler Medical University: 193 students (90 males, 103 females); Sulaimani University: 174 students (83 males, 91 females); and Duhok University: 91 students (46 males, 45 females).

Ethical approval was obtained from the Ethical Committee/College of Dentistry/University of Sulaimani. Students were informed about the study and assured of their anonymity. The close-ended self-administered validated questionnaire was prepared in English and consisted of three parts:

1. Part one related to sociodemographic characteristics of the study participants including gender, age, university, and stage
2. Part two consisted of 16 questions to determine the level of knowledge among dental students regarding HBV, its transmission, and prevention. The answer format for all the knowledge questions was Yes or No
3. Part three consisted of 10 questions about safety precautions regarding HBV. The answers were again in Yes or No format

### 2.1. Study Sample

All 458 dental students in the study population were invited to participate in this voluntary study. No sampling technique was employed as it was feasible to include the total study population. Dental students in the third, fourth, and fifth stages at Hawler Medical, Sulaimani, and Duhok universities who agreed to participate were included in the study, but incomplete questionnaires were excluded from consideration.

### 2.2. Data Collection

The questionnaires were distributed in the lecture halls and were collected after 20 minutes by the researcher from 22 February to 23 March 2014.

The knowledge score for each individual was calculated by assigning a score of “1” for each “Yes” response to items (1, 2, 4, 5, 6, 7, 10, 12, 14, 16) and a score of “1” for each (No) response to items (3, 8, 9, 11, 13, 15). The safety precautions score for each individual was calculated by assigning a score of “1” for each “Yes” response to items (2, 4, 5, 6, 7, 9, 10) and a score of “1” again for each “No” response to items (1, 3, 8).

Scores for knowledge questions (1-16) were added together to obtain a total knowledge score for each individual. The mean knowledge score was calculated by dividing the total knowledge scores of all individuals by the number of individuals. As this study was investigating general knowledge of HBV, the students were divided into three groups: weak (score of ≤4), intermediate (score of 5-8), and good (score of ≥9). Regarding safety precautions level, they were divided into weak (score of ≤3), intermediate (score of 3-6), and good (score of ≥7).

### 2.3. Statistical Analysis

Descriptive statistics were used to measure the mean and standard deviation (SD), and a chi-square test was conducted to compare categorical variables. Analysis of variance (ANOVA) was used to compare the mean of knowledge and safety precaution scores across Sulaimani, Hawler Medical, and Duhok universities. A *p* value of ≤0.05 was considered significant for statistical analysis. Data analysis was conducted using the statistical software package IBMSPSS (Statistical Package for the Social Sciences version 22.0, Chicago IL, USA).

## 3. Results

Out of 458 dental students from Sulaimani, Hawler Medical, and Duhok universities invited to participate in the study, 372 returned fully completed questionnaires, giving a response rate of 81.2%. The mean age of the participants (females [52.2%] and males [47.8%]) was 21.77 ± 1.31. The demographic data are shown in Table 1.

### 3.1. Knowledge about Hepatitis B Virus Infection

Kurdistan dental college students demonstrated awareness about most of the questions directed to them, specifically regarding the following: types of hepatitis virus, life-threatening nature of the infection, preventable nature of the disease, the dental team being more prone to infection, and others. For most of the questions, no differences were identified between students from different universities. However, approximately 70.4% of the Hawler respondents considered physical contact as a risk factor for HVB infection when asked about the spreading mode of HBV, followed by 63.3% of Duhok and 44% of Sulaimani respondents, which amounted to a statistically significant difference (*p* = 0.001). In total, about 72.6% of respondents reported that HBV infection is transmitted by saliva, and 78.8% identified transmission by needle sharing. No significant differences between the three universities were found in regard to this question. This survey showed that 79.3% of Hawler respondents knew that chronic HBV infection confers a high risk of cirrhosis, followed by Duhok (83.5%) and then Sulaimani (68.1%) respondents, reflecting a statistically significant difference (*p* = 0.001) (Table 2).

In terms of knowledge about preventive measures, 91.9% correctly identified careful blood transfusion, 79.8% identified vaccination, and 75.3% identified legal sex as steps for preventing HBV infection. Regarding the respondents' knowledge about liver cancer, HBV was mentioned as a cause by 77.4%, with a statistically significant difference between the different universities (*p* = 0.014), i.e., the highest proportion (84.9%) of correct responses came from dental students of Hawler Medical University, followed by Duhok (74.7%) and Sulaimani **(**70.9%), as demonstrated in Table 2.

### 3.2. Safety Precautions regarding Hepatitis B Virus

Overall, the respondents had excellent knowledge of safety precautions including washing hands prior to and after treatment procedure, after exposure to a patient's body fluid, and wearing protective face masks. A significant difference was noted among dental students of Sulaimani, Hawler Medical, and Duhok universities in relation to checking the patient's blood tests for contagious diseases before dental procedures (*p* = 0.018). Furthermore, 81.6% of Sulaimani respondents, followed by 78.5% of Duhok and 65.1% of Hawler Medical respondents, confirmed that they checked the indicator showing whether or not instruments have been sterilized, with statistically significant differences (*p* = 0004). Among the respondents as a whole, wearing gloves, washing hands, using protective gowns, and protective masks as safety precautions were reported by 90.1%, 93.5%, 82.8%, and 96.0%, respectively. In addition, 71.2% said that they wore goggles and 70.4% reported bending needles after injections and discarding them in a medical waste container (Table 3).

### 3.3. Comparison of Respondents' Mean Knowledge and Safety Precautions Scores

The mean knowledge and safety precautions scores of the respondent dental students in Sulaimani, Hawler Medical, and Duhok universities were compared by means of the ANOVA test (Table 4). The mean knowledge score for the total study sample was 13.1 out of 16. Hawler Medical recorded a statistically significantly higher mean knowledge score than Sulaimani and Duhok Universities (*p* = 0.012). The mean score on safety precautions for the total sample was 8.0 out of 10. Duhok achieved a higher mean safety precautions score than Sulaimani and Hawler Medical universities, but the difference was not statistically significant (*p* = 0.222), as shown in Table 4.

## 4. Discussion

It is crucial for dental students to have sound knowledge about the hepatitis B Virus infection since the high occupational risk of this infection among medical and dental workers is well known, especially during the professional training period. Nowadays, following the emergence of COVID-19, dental students have encountered changes in the teaching format. Several containment measures have been applied to stop the pandemic contagion of the virus, including isolation, contact tracing and quarantine, physical distancing, hygiene measures, and lockdown [11, 13, 14].

This risk provides one of the major reasons for delivering knowledge about preventive measures and universal precautions. The mean knowledge score of the dental student respondents in the Kurdistan region (regarding Hepatitis B Virus, its transmission, and prevention) was 13.1, while the corresponding score for safety precautions was 8.0, which implies sound knowledge and positive behavior toward this infection and implementation of universal precautions.

The current research found that Hawler Medical recorded a higher mean knowledge score than Sulaimani and Duhok universities, a potential reason being that Hawler Medical University had the highest number of respondents. A similar study, conducted at Sultan Qaboos University in Sultanate of Oman, reported that the majority of the respondent students (75%) were aware that HBV is a common cause of hepatitis and 50.7% of them thought that HBV infection is preventable. Approximately 70% of them believed that screening blood for HBV renders blood safe for transfusion [15]. This result is in agreement with the present study.

In another previous study, conducted by Othman et al. in 2013 on dental students at Hawler Medical University to determine the students' level of knowledge about HBV, a high percentage of respondents (41%) showed poor knowledge about HBV and method of transmission. In contrast, the current study revealed that Hawler Medical University respondents recorded a higher mean knowledge score than those from Sulaimani and Duhok universities. This result indicates that since the previous study was conducted, students' knowledge levels and awareness regarding contagious and blood-borne diseases have improved at Hawler Medical University. Students have apparently become more acquainted with HBV, its methods of transmission, and the preventive measures required to stay safe from infection with HBV and other contagious diseases. Another explanation for the higher level of knowledge among Hawler Medical University respondents in the current study is that the sample size was larger than in the previous study. The small sample size and the fact that the respondents were drawn only from Hawler city may have made it difficult to detect factors with a statistically significant association with students' knowledge levels [16].

Several recent studies also recorded unsatisfactory findings related to dental students' knowledge, attitudes, and behavior regarding HVB, and all these studies suggested the necessity of conducting mandatory continuous health education courses among healthcare providers, including dental students, and involving social media, to spread the key messages regarding transmission and prevention of HBV alongside conventional educational courses for healthcare providers [17–19]. For example, A study by Eisa et al. [20], conducted among first-year medical sciences students in Jazan University, Saudi Arabia, reported only moderate (57.1%) mean knowledge of the mode of transmission among the respondents. The reported mean percentage of positive beliefs and attitudes of 40.4% reflects a poor attitude regarding HBV [20]. As the study was conducted on first-year students, a low level of knowledge among those students was to be expected. The study outcome reinforces calls for the provision of intensive courses about the transmission of infectious and blood-borne diseases among medical staff and as part of rigorous educational and training programs on infection control measures for students prior to graduation [21]. However, other studies have reported adequate knowledge among dental students, with proper implementation of standard infection control measures in dental practice, suggesting that a higher knowledge level among dental students plays a major role in establishing the right attitudes and practices [12, 22]. The above-discussed results reveal differences among dental students regarding their knowledge, attitude, and awareness about the hazard of HBV and risk of transmission and spread among the community. This is linked to variation in the level of education and standards of teaching in these universities, with the majority of data obtained from developing countries and those showing good responses indicating a higher level of education at their universities.

Although the large sample size is considered a point of strength of the current study, the study had some limitations. First, the close-ended type of questioning could not reveal exact details of the respondents' knowledge and practice. Furthermore, the current study was conducted among dental students alone without including other dental care providers such as dental assistants and other teaching staff that play a major role in the effective implementation of infection control methods.

HBV is a worldwide healthcare problem, with oral healthcare providers at especially high risk of infection. HBV is a blood-borne virus that can be transmitted in dental practice by contaminated instruments and via percutaneous and mucocutaneous exposure to saliva and blood of infected patients. Healthcare workers in general and oral healthcare providers, in particular, are continuously exposed to infected fluids from the oral cavity and are at a high risk of contracting and transmitting this virus. Since all other oral healthcare providers, such as hygienists and dental assistants and other teaching staff, as well as dental students, are involved in controlling infection of HBV, it is suggested that all oral care providers in dentistry colleges need to participate, along with dental students and teaching staff, in a wider study to provide further details about their role in the transmission and/or prevention of HBV in Kurdistan region.

Results of the current study showed a need to further improve knowledge and practice of protection among dental students and to raise levels of awareness regarding the transmission of HBV among the students and patients during their daily practice of dentistry tasks, in addition, to conduct mandatory vaccination programs for the students and other staff in contact with the patients. Furthermore, there needs to be greater emphasis on certain areas of transmission of HBV and safety precautions such as checking patients' blood test results before dental procedures.

Recently with the emergence of COVID-19 pandemic worldwide, dentistry is considered a transmission source of HBV, HIV, and COVID-19. Despite the acceptable level knowledge of protection, transmission, and spread of infectious diseases, increasing knowledge and raising students' perception are required particularly in dental schools by the authorized university staff by adding further preventive modules to the preclinical learning courses. Furthermore, the dentists' attitudes and practices toward using personal protection equipment have changes dramatically in recent years due to the COVID-19 pandemic. In Iraq, a study indicated that the dentists had satisfactory levels of practices and positive attitudes toward using personal protection equipment [23]. Thus, the changes in attitude and practice toward HBV infection need further investigation.

It is important to acknowledge that some differences were identified between Hawler Medical, Sulaimani, and Duhok universities which may be related to their educational and training programs. The students' knowledge can be further enhanced by adopting continuous dental education programs, seminars, and workshops about hepatitis B infection at the institutional level as “awareness is empowering.” It is suggested that a separate study should be conducted on the curricula and vaccination policies of the medical/dental colleges, and finally, a program of complete vaccination and health education is recommended for all first-year students in all allied health colleges in our region.

## 5. Conclusions

The present study concluded that the majority of the respondents are aware of HBV, its mode of transmission, infection, complications, vaccination, and safety precaution measures to prevent the spreading of the HBV. Moreover, these dental students feel that it is very important that dentists, dental auxiliaries, students, and patients are immunized against HBV. Despite the level of knowledge of HBV and use of safety precautions among the dental students in the Kurdistan region of Iraq being generally acceptable, some differences were identified between the three universities, Hawler Medical, Sulaimani, and Duhok, which may be related to variations in their educational and training programs.

## Figures and Tables

**Table 1:** Sociodemographic distribution of the study participants.

Characteristic		Frequency	Percentage
Gender	Male	178	47.8
	Female	194	52.2

University	Sulaimani	141	37.9
	Hawler medical	152	40.9
	Duhok	79	21.2

Stage	Third	129	34.7
	Fourth	140	37.6
	Fifth	103	27.7

**Table 2:** Correct responses regarding HBV knowledge across the participating universities.

No	Questions regarding knowledge	University						Total (%)	Chi-square value	*p* value
		Sulaimani		Hawler medical		Duhok				
		No.	%	No.	%	No.	%			
1	Do you have heard about hepatitis B virus?	139	98.6	147	96.7	78	98.7	97.8	1.590	0.4
2	Is infection with HBV symptomatic?	111	78.7	122	80.3	59	74.7	78.5	0.966	0.6
3	Is infection with HBV temporary?	111	78.7	123	80.9	57	72.2	78.2	2.380	0.3
4	Can HBV infection be prevented?	121	85.5	137	90.1	72	91.1	88.7	1.952	0.3
5	Is HBV a life-threatening infection?	127	90.1	140	92.1	71	89.9	90.9	0.482	0.7
6	Are dentists and dental assistants more susceptible to HBV infection through cross-infection?	137	97.2	148	97.4	73	92.4	96.2	4.074	0.1
7	Have you heard of additional types of hepatitis?	135	95.7	144	94.7	73	92.4	94.6	1.116	0.5
8	Is physical contact a method of HBV transmission?	62	44.0	107	70.4	50	63.3	58.9	21.901	0.001
9	Body fluid is not a method of transmission of hepatitis B?	99	70.2	113	74.3	58	73.4	72.6	0.662	0.7
10	Is saliva a method of HBV transmission?	118	83.7	114	75.0	65	82.3	79.8	3.801	0.1
11	Needle sharing is not a Mode of HBV transmission?	105	74.5	127	83.6	61	77.2	78.8	3.753	0.1
12	Is cautious blood transfusion a step to avoid the spread of HBV?	131	92.9	136	89.5	75	94.9	91.9	2.382	0.3
13	Vaccination is not a step to prevent HBV transmission?	110	78.0	122	80.3	65	82.3	79.8	0.601	0.7
14	Is legitimate sex a step to avoid the spread of HBV?	102	72.3	116	76.3	62	78.5	75.3	1.177	0.5
15	Chronic HBV infection does not cause cirrhosis	96	68.1	133	87.5	66	83.5	79.3	17.897	0.001
16	Does chronic HBV infection lead to liver cancer?	100	70.9	129	84.9	59	74.7	77.4	8.568	0.014

**Table 3:** Correct responses on safety precautions across the participating universities.

No	Questions regarding safety precautions	University						Total (%)	Chi-square value	*p* value
		Sulaimani		Hawler medical		Duhok				
		No.	%	No.	%	No.	%			
1	I do not wear gloves when I touch the patient's membranes or non-intact skin	122	86.5	142	93.4	71	89.9	90.1	3.887	0.143
2	I always wash my hands prior to and after each treatment procedure	128	90.8	147	96.7	73	92.4	93.5	4.48	0.106
3	I do not use goggles during treatment for the patients	98	69.5	113	74.3	54	68.4	71.2	1.242	0.537
4	I always wash my hands after touching patients' body fluids	132	93.6	142	93.4	73	92.4	93.3	0.127	0.939
5	I put on protective gowns to protect myself during treatment procedures	116	82.3	124	81.6	68	86.1	82.8	0.782	0.676
6	I use a protective mask to be safe when during treatment procedures	138	97.9	146	96.1	73	92.4	96.0	3.916	0.141
7	After each injection, I bend the needles and put them in a medical waste container	100	70.9	103	67.8	59	74.7	70.4	1.222	0.543
8	I do not examine the patient′s blood tests for contagious infections prior to a procedure	95	67.4	76	50.0	50	63.3	59.4	11.868	0.018
9	I check the indicator to see if the instruments have been sterilized prior to their use in a treatment procedure	115	81.6	99	65.1	62	78.5	74.2	11.274	0.004
10	I give information to my patients about hepatitis and offer vaccination to them	100	70.9	108	71.1	64	81.0	73.1	3.181	0.204

**Table 4:** Comparison of mean knowledge and safety precautions scores across the three universities.

Parameters	University	No.	*Mean* ± *SD*	Minimum score	Maximum score	*F* test	*p* value
Knowledge	Sulaimani	141	12.80 ± 2.12	6	16	4.471	**0.012**∗
	Hawler medical	152	13.52 ± 1.97	7	16		
	Duhok	79	13.17 ± 2.16	7	16		

Safety precautions	Sulaimani	141	8.11 ± 1.58	3	10	1.511	0.222
	Hawler medical	152	7.89 ± 1.74	3	10		
	Duhok	79	8.26 ± 1.40	4	10		

^∗^Statistically significant

## Data Availability

The raw data supporting the conclusions of this article will be made available by the authors, without undue reservation.
